This article has been retracted.

# Diagnosis of Microvascular Angina Using Cardiac Magnetic Resonance

**DOI:** 10.1016/j.jacc.2017.12.046

**Published:** 2018-03-06

**Authors:** Alexander Liu, Rohan S. Wijesurendra, Joanna M. Liu, John C. Forfar, Keith M. Channon, Michael Jerosch-Herold, Stefan K. Piechnik, Stefan Neubauer, Rajesh K. Kharbanda, Vanessa M. Ferreira

**Affiliations:** a Oxford Centre for Clinical Magnetic Resonance Research, Division of Cardiovascular Medicine, Radcliffe Department of Medicine, University of Oxford, Oxford, United Kingdom; b Oxford Heart Centre, John Radcliffe Hospital, Oxford, United Kingdom; c Division of Cardiovascular Medicine, Radcliffe Department of Medicine, University of Oxford, Oxford, United Kingdom; d Brigham and Women’s Hospital, Radiology, Cardiovascular Imaging, Boston, Massachusetts

**Keywords:** cardiac magnetic resonance, index of microcirculatory resistance, inducible ischemia, microvascular dysfunction, myocardial perfusion reserve index, AUC, area under the curve, CAD, coronary artery disease, CI, confidence interval, CMD, coronary microvascular dysfunction, CMR, cardiac magnetic resonance, FFR, fractional flow reserve, IMR, index of microcirculatory resistance, LGE, late gadolinium enhancement, MBF, myocardial blood flow, MPR, myocardial perfusion reserve, MPRI, myocardial perfusion reserve index, NOCAD, nonobstructive coronary artery disease, QCA, quantitative coronary angiography, ROC, receiver-operating characteristic

## Abstract

**Background:**

In patients with angina and nonobstructive coronary artery disease (NOCAD), confirming symptoms due to coronary microvascular dysfunction (CMD) remains challenging. Cardiac magnetic resonance (CMR) assesses myocardial perfusion with high spatial resolution and is widely used for diagnosing obstructive coronary artery disease (CAD).

**Objectives:**

The goal of this study was to validate CMR for diagnosing microvascular angina in patients with NOCAD, compared with patients with obstructive CAD and correlated to the index of microcirculatory resistance (IMR) during invasive coronary angiography.

**Methods:**

Fifty patients with angina (65 ± 9 years of age) and 20 age-matched healthy control subjects underwent adenosine stress CMR (1.5- and 3-T) to assess left ventricular function, inducible ischemia (myocardial perfusion reserve index [MPRI]; myocardial blood flow [MBF]), and infarction (late gadolinium enhancement). During subsequent angiography within 7 days, 28 patients had obstructive CAD (fractional flow reserve [FFR] ≤0.8) and 22 patients had NOCAD (FFR >0.8) who underwent 3-vessel IMR measurements.

**Results:**

In patients with NOCAD, myocardium with IMR <25 U had normal MPRI (1.9 ± 0.4 vs. controls 2.0 ± 0.3; p = 0.49); myocardium with IMR ≥25 U had significantly impaired MPRI, similar to ischemic myocardium downstream of obstructive CAD (1.2 ± 0.3 vs. 1.2 ± 0.4; p = 0.61). An MPRI of 1.4 accurately detected impaired perfusion related to CMD (IMR ≥25 U; FFR >0.8) (area under the curve: 0.90; specificity: 95%; sensitivity: 89%; p < 0.001). Impaired MPRI in patients with NOCAD was driven by impaired augmentation of MBF during stress, with normal resting MBF. Myocardium with FFR >0.8 and normal IMR (<25 U) still had blunted stress MBF, suggesting mild CMD, which was distinguishable from control subjects by using a stress MBF threshold of 2.3 ml/min/g with 100% positive predictive value.

**Conclusions:**

In angina patients with NOCAD, CMR can objectively and noninvasively assess microvascular angina. A CMR-based combined diagnostic pathway for both epicardial and microvascular CAD deserves further clinical validation.

In patients with angina, up to 90% have nonobstructive coronary artery disease (NOCAD), as shown in the recent PROMISE (Prospective Multicenter Imaging Study for Evaluation of Chest Pain) trial 1, 2. Although these patients with “microvascular angina” are often reassured as having a low risk for ischemic heart disease or empirically treated with antianginal medications, they experience reduced quality of life and adverse clinical outcomes and contribute to increased health care bills 1, 3, 4. Ischemia due to coronary microvascular dysfunction (CMD) remains a diagnostic challenge in general cardiology practice.

Currently, fractional flow reserve (FFR) is the invasive gold standard for assessing flow limitation across an epicardial coronary stenosis, but it does not assess the microcirculation (5). The index of microcirculatory resistance (IMR) is an invasive thermodilution-based marker of microvascular function (6) associated with microvascular obstruction and adverse prognosis after acute coronary occlusion 7, 8. In patients with stable angina and NOCAD, CMD can be identified by using an IMR threshold of ≥25 U 9, 10, and an elevated IMR is linked to lower Duke treadmill scores (10), with prognostic value in predicting long-term major adverse cardiac events (11). However, IMR can only be determined during invasive coronary angiography by experienced operators. Thus, being able to noninvasively and conveniently assess CMD is highly desirable for clinical risk stratification and guiding patient therapy.

Cardiac magnetic resonance (CMR) is an ideal noninvasive modality for assessing patients with angina 4, 12. Adenosine stress CMR evaluates myocardial perfusion with high spatial resolution and accurately detects ischemia due to obstructive epicardial CAD 13, 14. Although previous studies have evaluated myocardial perfusion in patients with NOCAD using CMR 15, 16, 17, these studies have included heterogeneous patient cohorts, without objective validation against an invasive marker of CMD; the result is conflicting findings with limited direct clinical applicability 15, 16, 17, 18. There is currently no accepted objective diagnostic threshold for assessing CMD using CMR.

The goal of the present study was to validate stress perfusion CMR to objectively and noninvasively diagnose microvascular angina, with correlation to invasive coronary measures (FFR and IMR). We also examined the underlying mechanism for impaired myocardial perfusion reserve (MPR) in CMD, using absolute quantification of myocardial blood flow (MBF) at rest and during adenosine stress, as validated against IMR.

## Methods

### Study population

Fifty patients with angina and suspected or known CAD referred for outpatient diagnostic coronary angiography were recruited for study. Patients underwent CMR scans at 2 commonly used clinical field-strengths: 1.5-T (n = 25; Magnetom Avanto; Siemens Healthcare GmbH, Erlangen, Germany) or 3-T (n = 25; Magnetom Trio, A Tim System; Siemens Healthcare GmbH). We also recruited 20 age-matched healthy control subjects (no cardiovascular disease, no regular medications, and normal electrocardiogram) to undergo CMR at 1.5-T (n = 10) and 3-T (n = 10) using the same CMR scanners and protocol as the study patients. Perfusion measures (myocardial perfusion reserve index [MPRI] and MBF) were comparable between the 1.5-T and 3-T scans in control subjects and patients (all p > 0.50).

All study procedures were approved by a local ethics committee (Reference: 13/SC/0376), and all subjects provided written informed consent.

### CMR protocol

All subjects abstained from caffeine for 24 h before the CMR. The CMR was performed by using established techniques, including cine, adenosine stress and rest perfusion, and late-gadolinium enhancement (LGE) imaging, as previously described (19) (Online Appendix). All subjects had good hemodynamic stress response (>10 beats/min increase in heart rate and ≥1 adenosine-related symptom [e.g., chest tightness]) (20). In addition, 60% (30 of 50) of patients and all control subjects had a significant (>10 mm Hg) drop in systolic blood pressure during stress.

### Invasive coronary angiography and physiology assessments

Within 7 days post-CMR, all 50 patients underwent invasive coronary angiography. Quantitative coronary angiography (QCA) was also performed offline by using Medcon QCA software (Medcon Ltd., Tel Aviv, Israel), as previously described (21).

FFR and IMR were measured, as described elsewhere (22) (Online Appendix), by operators blinded to the research CMR. IMR (distal coronary pressure × hyperemic mean transit time) was corrected by using the Yong formula to account for any effects of collateral circulation (23).

In total, 28 patients had significant epicardial CAD (≥50% visual angiographic stenosis; 23 with 1-vessel CAD, 3 with 2-vessel CAD, and 2 with 3-vessel CAD). In these patients, 86% of epicardial lesions (30 of 35 vessels) were functionally obstructive (FFR ≤0.8). The remaining 22 patients all had angiographic NOCAD (<50% visual stenosis), where 100% (66 of 66) of coronary arteries were FFR-negative (>0.8), and IMR was assessed in all 66 vessels.

### CMR image analysis

All CMR images were analyzed by using the commercially available cmr^42^ software (Circle Cardiovascular Imaging Inc., Calgary, Alberta, Canada) 19, 24. Myocardial perfusion images were analyzed as previously described (19), blinded to clinical information, other CMR, and invasive coronary data (Online Appendix). MPRI was derived semi-quantitatively (J.M.L.) as the stress/rest ratio of myocardial signal intensity upslopes, normalized to the arterial input function (19). Absolute quantification of MBF (in milliliters per minute per gram) was performed (A.L.) by using model-independent Fermi deconvolution of myocardial and arterial input signal intensity curves, as previously described (25).

To enable correlation between perfusion measures (MPRI and MBF) and invasive coronary measurements (FFR and IMR) on a per-vessel basis, myocardial perfusion images were segmented and allocated to each coronary artery territory according to the American Heart Association’s 16-segment model, accounting for coronary artery dominance (as described elsewhere [26]). Segmental MPRI and MBF values were then averaged for each coronary artery territory and matched to FFR and IMR data for further analysis. Left ventricular function and LGE imaging were analyzed as previously described (19).

### Statistical analysis

An optimal MPRI threshold for symptomatic inducible ischemia on stress perfusion CMR was first derived using the 28 patients with angina and obstructive epicardial CAD and the 20 normal control subjects. A receiver-operating characteristic (ROC) curve was used with myocardium downstream of FFR ≤0.8 vessels as true-positives for ischemia and normal controls as true-negatives. This MPRI threshold was then applied in 22 patients with 3-vessel NOCAD to determine its diagnostic performance for detecting significantly impaired perfusion due to CMD with high IMR.

All continuous variables were normally distributed, as checked by using the Kolmogorov-Smirnov test, and are expressed as mean ± SD. Each patient with 3-vessel NOCAD contributed 3 IMR values (total 66), and the intraclass correlation coefficient was calculated to determine the need to adjust the data for clustering (27). The intraclass correlation coefficient was very low for IMR (0.02; 95% CI: –0.09 to 0.12), indicating that the values were not strongly related within the same patient; the relations between IMR and CMR data were analyzed on a per-vessel basis. Due to the highly statistically significant comparisons observed throughout the study, we used a conservative approach to compensate for potential multiple comparisons and any remaining within-individual correlations of IMR data by reducing the threshold p value from the conventional 0.05 to 0.01. This approach likely overcompensates for the worst-case scenario of 3 fully dependent variables within the same individual. For all analyses, p values <0.01 were considered statistically significant.

Comparisons between 2 separate data groups were performed by using unpaired Student’s *t*-test. Comparisons between ≥3 separate data groups were performed by using analysis of variance with a Bonferroni post hoc method. Categorical data were compared by using the Fisher exact test. Correlations were assessed by using the Spearman’s rank correlation coefficients (rho). For ROC analysis, area under the curve (AUC) with 95% confidence intervals (CIs) are reported, as well as sensitivity, specificity, accuracy, positive predictive values, and negative predictive values where appropriate. All analyses were performed by using MedCalc version 12.7.8 (MedCalc Software, Ostend, Belgium).

## Results

### Subject characteristics

Subject characteristics are summarized in Table 1. The 28 patients with obstructive epicardial CAD contributed a total of 30 FFR-positive (mean FFR: 0.60; range: 0.28 to 0.79) coronary arteries to the analysis (Figure 1), which were also angiographically significant (75 ± 3% stenosis) on QCA. The 22 patients with NOCAD contributed a total of 66 FFR-negative vessels (mean FFR: 0.92; range: 0.80 to 1.00), with minimal angiographic disease (10 ± 5%) on QCA.

**Figure 1:** Study Flowchart Numbers represent either the number of patients or the number of coronary arteries, as indicated. CAD = coronary artery disease; CMR = cardiac magnetic resonance; FFR = fractional flow reserve; IMR = index of microcirculatory resistance; NOCAD = nonobstructive coronary artery disease.

**Table 1:** Subject Characteristics

	Normal Control Subjects (n = 20)	Patients With Obstructive CAD (n = 28)	Patients With All NOCAD (n = 22)	p Value
Age, yrs	61 ± 7	64 ± 9	65 ± 8	0.31
Body mass index, kg/m^2^	25 ± 5	28 ± 4	31 ± 5	0.07
Male	13 (65)	20 (71)	14 (64)	0.82
Angina characteristics				
CCS angina score	–	1.9 ± 0.6	1.9 ± 0.5	0.84
Diamond and Forrester score, %	–	57 (13–93)	56 (7–94)	0.89
Comorbidities				
Ex-smoker	0 (0)	16 (57)	13 (59)	0.98
Diabetes mellitus	0 (0)	6 (21)	8 (36)	0.34
Hypertension	0 (0)	13 (46)	13 (59)	0.41
Hyperlipidemia	0 (0)	15 (54)	10 (45)	0.78
Known CAD	–	15 (54)	0 (0)	<0.001
Previous PCI	–	7 (25)	0 (0)	<0.001
Previous CABG	–	0 (0)	0 (0)	–
Medications				
Aspirin	0 (0)	28 (100)	20 (91)	0.19
Beta-blocker	0 (0)	25 (89)	16 (72)	0.16
ACE inhibitors/ARBs	0 (0)	16 (57)	11 (50)	0.78
Statin	0 (0)	16 (57)	11 (50)	0.78
Nitrates	0 (0)	15 (54)	13 (59)	0.78
Nicorandil	0 (0)	3 (11)	4 (18)	0.68
Ranolazine	0 (0)	1 (4)	2 (9)	0.58
CMR hemodynamic data				
Resting heart rate, beats/min	63 ± 10	63 ± 14	65 ± 11	0.70
Stress heart rate, beats/min	90 ± 11	93 ± 10	89 ± 15	0.53
Rest SBP, mm Hg	135 ± 16	139 ± 31	141 ± 20	0.41
Stress SBP, mm Hg	130 ± 11	132 ± 17	130 ± 17	0.65
Resting RPP, beats/min ∙ mm Hg	9,200 ± 2,000	9,100 ± 2,600	9,200 ± 2,400	0.79
Stress RPP, beats/min∙ mm Hg	11,700 ± 2600	12,100 ± 3,200	11,800 ± 2,900	0.24

Values are mean ± SD, n (%), or mean (range). p values were determined by using an analysis of variance with a Bonferroni post hoc method for continuous variables and Fisher exact test for categorical variables.

ACE = angiotensin-converting enzyme; ARB = angiotensin receptor blocker; CABG = coronary artery bypass grafting; CAD = obstructive epicardial coronary artery disease; CCS = Canadian Cardiovascular Society; CMR = cardiac magnetic resonance; NOCAD = nonobstructive coronary artery disease; PCI = percutaneous coronary intervention; RPP = rate pressure product; SBP = systolic blood pressure.

Table 2 presents a summary of coronary physiology measures. In patients with NOCAD, IMR was not significantly affected by the Yong formula corrections (23) (IMR before correction: 27 ± 14 U vs. IMR after correction 27 ± 14 U; paired p = 0.30), suggesting minimal influence from collateral circulations. IMR was not significantly correlated to FFR (rho = 0.07; p = 0.59).

**Table 2:** Coronary Physiology and CMR Parameters

	Normal Control Subjects (n = 20)	Patients With Obstructive CAD (n = 28)	Patients With All NOCAD (n = 22)	p Value
CMR parameters				
LV EDVi, ml/m^2^	75 ± 11	78 ± 11	77 ± 13	0.40
LV ESVi, ml/m^2^	28 ± 8	32 ± 12	30 ± 12	0.26
LV SVi, ml/m^2^	47 ± 6	46 ± 10	47 ± 12	0.91
LV ejection fraction, %	62 ± 5	59 ± 9	61 ± 10	0.35
LV mass index, g/m^2^	58 ± 10	59 ± 11	56 ± 13	0.25
Mean LV wall_thickness_, mm	7.9 ± 0.6	7.5 ± 1.5	7.4 ± 0.7	0.23
MPRI	2.0 ± 0.3	1.2 ± 0.4∗	1.6 ± 0.5∗†	<0.001
Rest MBF	1.1 ± 0.2	1.1 ± 0.3	1.1 ± 0.2	0.80
Stress MBF	3.0 ± 0.5	1.4 ± 0.4∗	2.1 ± 0.8∗†	<0.001
LGE, %	0 ± 0	10 ± 5∗	0 ± 0†	<0.001
Coronary physiology				
FFR	–	0.60 (0.28–0.79)	0.92 (0.80–1.00)	<0.001
IMR, U	–	27 ± 15	27 ± 14	0.91
IMR_corr_, U	–	21 ± 11	27 ± 14	0.05
Distribution of FFR and IMR				
Total vessels assessed	–	60 (71)	66 (100)	0.17
FFR <0.8 and IMR ≥25 U	–	10 (17)	0 (0)	<0.001
FFR <0.8 and IMR <25 U	–	20 (33)	0 (0)	<0.001
FFR ≥0.8 and IMR ≥25 U	–	11 (18)	28 (42)	<0.001
FFR ≥0.8 and IMR <25 U	–	19 (32)	38 (58)	<0.001

Values are mean ± SD, mean (range), or n (%). All p values for CMR parameters were determined by using an analysis of variance with Bonferroni post hoc method. All p values for coronary physiology were determined by using an unpaired Student’s *t*-test.

EDVi = end-diastolic volume index; ESVi = end-systolic volume index; FFR = fractional flow reserve; IMR = index of microvascular resistance; IMR_corr_ = Yong formula–corrected IMR; LGE = late gadolinium enhancement; LV = left ventricular; MBF = myocardial blood flow; MPRI = myocardial perfusion reserve index; SVi = stroke volume index; other abbreviations as in Table 1.

∗ p < 0.01 compared with control subjects.

† p < 0.01 compared with patients with CAD.

Myocardial infarct scars were detected in 4 of 28 patients with obstructive CAD on CMR LGE imaging (all <50% transmurality). Patients with NOCAD and control subjects had no scars on LGE. To present a true representation of myocardial perfusion in noninfarcted myocardium, segments with scars were excluded. This method did not lead to exclusion of any patients.

### Patterns of MPRI in control subjects and patients with obstructive CAD and NOCAD

As a reference, myocardium downstream of obstructive CAD (FFR ≤0.8) had significantly lower MPRI than control subjects (1.2 ± 0.4 vs. 2.0 ± 0.3; p < 0.001). Downstream of NOCAD (FFR >0.8) vessels, MPRI correlated significantly with IMR (rho = –0.67; p < 0.001) (Figure 2) and coronary flow reserve (rho = 0.41; p < 0.001) (Online Figure 1) but not with FFR (rho = 0.04; p = 0.48).

**Figure 2:** Relations Between MPRI and IMR in Patients With Angina and NOCAD Each **dot** represents data from a single vessel (66 vessels from 22 patients with NOCAD). Rho is the Spearman’s correlation coefficient. MPRI = myocardial perfusion reserve index; other abbreviations as in Figure 1.

CMD was defined as myocardium with IMR ≥25 U downstream of NOCAD (FFR >0.8) vessels, as previously described (28). Myocardium with IMR <25 U had similar MPRI compared with normal control subjects (1.9 ± 0.4 vs. 2.0 ± 0.3; p = 0.49) (Figure 3A). In contrast, myocardium with IMR ≥25 U had impaired MPRI (1.2 ± 0.3), similar to myocardium downstream of obstructive (FFR ≤0.8) CAD in patients with angina (1.2 ± 0.3 vs. 1.2 ± 0.4; p = 0.61).

**Figure 3:** Patterns of MPRI in Normal Control Subjects and Patients With Obstructive CAD and Patients With All NOCAD **(A)** Myocardium downstream FFR >0.8 vessels with IMR <25 U (38 vessel territories in 17 patients) had MPRI similar to control subjects; myocardium downstream FFR >0.8 vessels with IMR ≥25 U (28 vessel territories in 15 patients) had impaired MPRI, similar to downstream obstructive (FFR ≤0.8) epicardial CAD (30 vessel territories in 28 patients). **(B)** The diagnostic performance of MPRI in patients with all NOCAD (66 vessel territories in 22 patients) for detecting ischemia related to coronary microvascular dysfunction (FFR >0.8 and IMR ≥25 U). All bars represent mean ± 1 SD. Area under the curve, p < 0.0001. Brackets include 95% confidence intervals. *p < 0.01; NS denotes p > 0.10. Abbreviations as in Figures 1 and 2.

### MPRI thresholds for assessing microvascular inducible ischemia

An MPRI threshold of 1.4 was optimal for detecting inducible myocardial ischemia from obstructive (FFR ≤0.8) CAD (AUC: 0.95; 95% CI: 0.85 to 0.99; p < 0.001). Myocardium downstream of obstructive (FFR ≤0.8) CAD served as true-positives; normal myocardium of control subjects served as true-negatives.

This threshold for inducible ischemia was then applied to patients with 3-vessel NOCAD. The MPRI threshold of 1.4 also accurately detected inducible ischemia due to CMD (IMR ≥25 U) (AUC: 0.90; 95% CI: 0.80 to 0.96; p < 0.0001), with a specificity of 95% (95% CI: 82% to 99%), a sensitivity of 89% (95% CI: 78% to 98%), and accuracy of 92% (95% CI: 80% to 99%) (Figure 3B). An MPRI threshold of 1.6 yielded a high negative predictive value (95%; 95% CI: 79% to 99%) and sensitivity (94%; 95% CI: 77% to 99%) for ruling out significant inducible ischemia due to CMD.

Downstream of nonobstructive FFR ≥0.8 coronary arteries in patients with obstructive CAD (30 vessels), the same MPRI threshold of 1.4 also accurately detected CMD (IMR ≥25 U) (AUC: 0.89; 95% CI: 0.81 to 0.96; p < 0.001).

### Patterns of MBF in control subjects and patients with obstructive CAD and NOCAD

To further understand the impaired MPRI observed in NOCAD, absolute quantification of MBF was performed at rest and during stress. Resting MBF was similar between normal control subjects, myocardium downstream of epicardial CAD, myocardium downstream of NOCAD with IMR <25 U and myocardium downstream of NOCAD with IMR ≥25 U, p = 0.76 (Figure 4A).

**Figure 4:** MBF Patterns in Patients and Control Subjects Patterns of myocardial blood flow (MBF) **(A)** at rest, **(B)** during adenosine stress, and **(C)** myocardial perfusion reserve (MPR: stress MBF / rest MBF) in normal control subjects and patients. The number of patients and vessel territories are as per Figure 3. All bars represent mean ± SD. *p < 0.01; NS denotes p > 0.10. Other abbreviations as in Figure 1.

During adenosine stress, myocardium downstream of obstructive epicardial CAD (FFR ≤0.8) had significantly lower stress MBF than normal control subjects (1.4 ± 0.4 ml/min/g vs. 3.0 ± 0.5 ml/min/g; p < 0.0001) (Figure 4B). Downstream of NOCAD (FFR >0.8), myocardium with IMR ≥25 U had a similar degree of impairment in stress MBF as myocardium downstream of obstructive epicardial CAD (1.5 ± 0.4 ml/min/g vs. 1.4 ± 0.4 ml/min/g; p = 0.14). Interestingly, although myocardium with IMR <25 U had higher stress MBF (2.6 ± 0.7 ml/min/g) than both myocardium with IMR ≥25 U (1.5 ± 0.4 ml/min/g) and myocardium downstream of obstructive CAD (1.4 ± 0.4 ml/min/g; all p < 0.001), it was still significantly blunted compared with that of healthy age-matched control subjects (2.6 ± 0.7 ml/min/g vs. 3.0 ± 0.5 ml/min/g; p < 0.01).

The quantitatively derived MPR (stress MBF / resting MBF) showed a similar pattern as for semi-quantitatively derived MPRI (Figure 4C). On ROC analysis, semi-quantitative MPRI, quantitative MPR (stress MBF / resting MBF), and stress MBF alone all had similar diagnostic performance for detecting impaired perfusion due to CMD (IMR ≥25 U) (AUC 0.90 vs. AUC 0.87 vs. AUC 0.91, respectively; all comparisons p > 0.70). Figure 5 presents the assessment of a patient with microvascular angina using CMR MPRI.

**Figure 5:** Assessment of Microvascular Inducible Ischemia Using CMR This 68-year-old male patient with angina had a normal resting electrocardiogram, and an exercise electrocardiogram was aborted early due to severe angina. A single photon-emission computed tomography scan was negative for inducible ischemia, and dobutamine stress echocardiography showed possible inferior wall hypokinesia during stress. He was referred for invasive coronary angiography. On 3-T CMR pre-angiography (normal ejection fraction: 60%; no regional wall motion abnormalities), the patient had no obvious regional reversible perfusion defects, and no myocardial infarction on late gadolinium enhancement (LGE) imaging, suggesting no obstructive epicardial CAD. However, the MPRI was globally impaired (<1.4), corresponding to 3 nonobstructive coronary arteries with elevated IMR (>25 U) on invasive angiography. This case shows that CMR may provide an objective one-stop assessment of microvascular ischemia, potentially avoiding multiple tests and invasive procedures. LAD = left anterior descending artery; LCx = left circumflex artery; RCA = right coronary artery; other abbreviations as in Figures 1 and 2.

### Identification of subtle deficits in stress MBF in patients with NOCAD

In patients with NOCAD (FFR >0.8) and normal IMR (<25 U) but blunted stress MBF compared with control subjects (Figure 4B), stress MBF was not significantly correlated to IMR (range: 10 to 25 U; rho = 0.09; p = 0.58). This impaired augmentation of stress MBF suggests possible mild or early CMD, insensitive to detection with the use of ratio-based measures (MPRI and quantitative MPR). A stress MBF threshold of 2.3 ml/min/g distinguished this mild CMD from normal control subjects with 100% specificity (95% CI: 83% to 100%) and 100% positive predictive value (95% CI: 81% to 100%), (AUC 0.76; 95% CI: 0.63 to 0.86; p < 0.0001).

## Discussion

The present study used adenosine stress CMR to objectively assess inducible ischemia due to CMD in patients with angina and NOCAD, as validated against the IMR. Impairments in MPR due to CMD (IMR ≥25 U) were driven by blunted augmentation of hyperemic MBF and were comparable to ischemic myocardium downstream of FFR-positive obstructive CAD (5). An MPRI threshold of 1.4 accurately detected significant CMD-related hypoperfusion. Furthermore, a quantitatively derived stress MBF threshold of 2.3 ml/min/g can detect mild CMD. Integration of MPRI and MBF assessment into the clinical CMR workflow can provide a noninvasive approach for evaluating both epicardial and microvascular CAD in patients with angina (Central Illustration), which deserves further validation in an all-comers population.

**Central Illustration:** Clinical Diagnostic Pathway Using CMR for Epicardial and Microvascular CAD A potential integrated clinical pathway for diagnosing both epicardial and microvascular coronary artery disease (CAD) using noninvasive cardiac magnetic resonance (CMR). Using this pathway, patients with obstructive epicardial CAD can be diagnosed on stress perfusion CMR according to conventional visual assessment. Patients without significant visual perfusion defect on CMR can undergo semi-quantitative myocardial perfusion reserve index (MPRI) assessment for microvascular CAD. Patients with an MPRI <1.4 have a high likelihood of having significant microvascular CAD; an MPRI >1.6 makes this diagnosis unlikely. For patients with an MPRI between 1.4 and 1.6, more detailed assessment of stress myocardial blood flow (MBF) can enable the detection of milder forms of microvascular CAD.

### Microvascular inducible ischemia is challenging to detect visually

In stress perfusion CMR, obstructive epicardial CAD leads to regional perfusion defects that can be visually distinguished from areas without perfusion defects. In the absence of obstructive epicardial CAD, CMD may also induce myocardial hypoperfusion, but this process rarely results in regional or global perfusion defects that can be assessed visually. Furthermore, qualitative assessment of hypoperfusion as a binary “yes/no” output cannot inform about the severity or the distribution of microvascular disease.

Advances in CMR image post-processing methods enabled detailed examination of MPR and MBF, which are well validated for detecting obstructive CAD 13, 29, 30. However, because visual assessment of perfusion images is already accurate for detecting obstructive CAD in routine clinical workflow, these more sophisticated post-processing methods have largely remained in the realm of research. For detecting microvascular inducible ischemia, however, these more advanced methods are invaluable because visual assessment is not possible.

In previous studies, microvascular ischemia has largely been a diagnosis of exclusion, rather than being objectively demonstrated 15, 16, 17, due to either the complete lack of validation against invasive reference standards for CMD 15, 16, 18 or validation against invasive markers that are not specific for the microcirculation, such as coronary flow reserve or coronary reactivity testing (17). Moreover, nonobstructive coronary arteries in previous studies were defined according to angiographic appearances alone 12, 15, 16, 17, 18, which informs little about their physiological significance. This limitation of previous studies introduces disease heterogeneities, leading to conflicting results 15, 16, 17, 18, which render the derivation of objective diagnostic thresholds highly challenging thus far.

### Microvascular ischemia detection

As a representative threshold for inducible ischemia, an MPRI cutoff based on myocardium downstream of obstructive epicardial CAD was established, defined using the clinically accepted FFR (≤0.8) method (5). This threshold (MPRI 1.4) then accurately detected significantly impaired myocardial perfusion due to CMD in a separate group of patients with angiographically and physiologically (FFR >0.8) nonobstructive coronary arteries, as referenced to invasive IMR. In this way, we adjudicated that myocardial perfusion deficits were related to an invasive marker of CMD, enabling the derivation of an objective threshold on CMR for diagnosing microvascular ischemia.

The impaired MPR downstream of NOCAD with high IMR (≥25 U) being similar to downstream FFR ≤0.8 CAD supports the presence of microvascular inducible ischemia that could account for angina symptoms. This perfusion reserve impairment was driven by blunted hyperemic MBF, with normal resting MBF, indicating a functional vasodilatory deficit, despite achieving good hemodynamic response to adenosine stress in all these patients. Overall, it would seem that when myocardial perfusion becomes significantly impaired (MPRI <1.4), symptoms of angina would ensue, whether this outcome is due to obstructive epicardial CAD or coronary microvascular dysfunction.

Intriguingly, myocardium without significant epicardial CAD (FFR >0.8) or CMD (IMR <25 U) still had blunted stress MBF compared with that of normal control subjects. Here, CMR detects changes in MBF and may be sensitive to early or mild changes in CMD. Furthermore, this possible mild CMD in patients with stable angina was insensitive to detection with the use of ratio-based measures such as MPRI or quantitative MPR, which remained indistinguishable from normal (possibly due to the subtle nature of the findings). The underlying mechanisms for this observation, including structural (e.g., microvascular rarefaction) and/or functional (e.g., vasodilatory hyporeactivity) abnormalities, deserve further investigation. Absolute quantification of MBF represents a strength of CMR in the comprehensive, noninvasive assessment of these patients.

CMD is classically described as a global phenomenon across the myocardium (3). Although this description is consistent with our results in patients with NOCAD and 3-vessel high IMR (≥25 U) who had globally impaired MPRI with little regional variations, approximately one-half of our patients with NOCAD had a combination of vessels with high IMR and vessels with normal IMR. This interesting finding revealed a coronary-specific distribution of microvascular dysfunction in some patients; in fact, as the number of vessels with high IMR increased in each patient, there was progressive worsening of the global MPRI. This outcome may explain the heterogeneities in myocardial perfusion seen in previous studies, in which patients with angiographic NOCAD but varying distribution of CMD may have been studied 15, 16, 17. Clinically, the knowledge of single-vessel versus multivessel CMD may offer better risk stratification and disease monitoring tailored to the individual patient. This concept deserves further investigation.

### Clinical potential of CMR-based assessment of epicardial and microvascular CAD

Because stress perfusion CMR is excellent for ruling out obstructive epicardial CAD (31), integration of MPRI assessment may enable a dual evaluation of epicardial CAD (visual analysis) and microvascular dysfunction (MPRI/MBF) in a single CMR scan (Central Illustration). MPRI can be assessed by using commercially available software for direct clinical application, and stress MBF may enable the detection of subtle microvascular dysfunction, when the post-processing methods become available beyond experienced centers 12, 25. The prognostic implications of these approaches and their roles in guiding clinical management of patients with angina are the subject of active research.

There are 3 major clinical dilemmas surrounding patients with angina and NOCAD. First, objectively diagnosing microvascular angina is challenging due to the lack of noninvasive reference standard tests in clinical practice (4). Second, even when the clinical suspicion of microvascular angina is high, the clinician is hampered by a limited armamentarium of disease-modifying therapies for CMD. Patients are therefore either started empirically on antianginal medications or not treated at all. Third, there is currently a lack of objective methods for disease monitoring; hence, the true natural history of CMD progression in the clinical arena remains unclear. Objective diagnostic thresholds using CMR (or IMR) can offer patients with microvascular angina an objective explanation for their symptoms, which can improve psychological well-being. For clinicians, these markers may allow them to provide a more confident diagnosis for the patient, a firmer indication for commencing medical therapy, and potentiate the development and testing of novel therapies for microvascular ischemia. In addition to monitoring the changes in symptoms over time, which can be subjective, MPRI may provide an objective disease-monitoring tool in patients with angina and NOCAD. The prognostic values of MPRI and MPRI-guided therapy are important topics of active ongoing research.

### Study limitations and future directions

This study was conducted in a single tertiary-care center with a relatively small number of patients with NOCAD, although the 3-vessel assessment of coronary physiology (IMR and FFR) with matching multiparametric CMR data is unique. Admittedly, there is currently no true “gold standard” marker for myocardial ischemia, and this fact remains a limitation of most similar studies. In this study, CMR was chosen due to its high spatial resolution for assessing myocardial perfusion, and IMR was used as a reproducible invasive marker for CMD (28). The combination of high IMR ≥25 U and impaired MPRI, similar to downstream of significant FFR-positive epicardial CAD, strongly supported the presence of microvascular inducible ischemia in patients with NOCAD. Although CMR perfusion imaging achieved high diagnostic performance for diagnosing microvascular ischemia in this study, a CMR-based comprehensive diagnostic pathway that enables pre-angiography clinical decision-making in patients with angina and NOCAD deserves further validation in a larger prospective study. Future studies using position emission tomography and advanced metabolic imaging (e.g., hyperpolarized CMR imaging [32]), as well as other invasive methods (e.g., Doppler wire–based techniques), may be further informative for defining cellular myocardial ischemia in the context of CMD.

## Conclusions

In angina patients with NOCAD, CMR can objectively and noninvasively assess microvascular angina. A CMR-based combined diagnostic pathway for both epicardial and microvascular CAD deserves further clinical validation.

Perspectives **COMPETENCY IN PATIENT CARE AND PROCEDURAL SKILLS:** In patients with angina and nonobstructive coronary atherosclerosis (FFR >0.8), stress CMR can diagnose microvascular angina in viable myocardium using an MPRI threshold of 1.4, as validated against an elevated invasive IMR (≥25 U). The degree of impaired perfusion is similar to that in patients with angina due to obstructive CAD.

**TRANSLATIONAL OUTLOOK:** Further research is required to determine the prognostic implications of MPRI thresholds to guide therapy and monitor patients for coronary microvascular dysfunction.
